# Design of Intelligent Diagnosis and Treatment System for Ophthalmic Diseases Based on Deep Neural Network Model

**DOI:** 10.1155/2022/4934190

**Published:** 2022-07-05

**Authors:** Huihui Zhou

**Affiliations:** Taizhou Hospital of Zhejiang Province Affiliated to Wenzhou Medical University, Taizhou, Zhejiang 317099, China

## Abstract

Artificial intelligence (AI) has developed rapidly in the field of ophthalmology. Fundus images have become a research hotspot because they are easy to obtain and rich in biological information. The application of fundus image analysis (AI) in background image analysis has been deepened and expanded. At present, a variety of AI studies have been carried out in the clinical screening, diagnosis, and prognosis of eye diseases, and the research results have been gradually applied to clinical practice. The application of AI in fundus image analysis will improve the situation of lack of medical resources and low diagnosis efficiency. In the future, the research of AI eye images should focus on the comprehensive intelligent diagnosis of various ophthalmic diseases and complex diseases. The focus is to integrate standardized and high-quality data resources, improve algorithm efficiency, and formulate corresponding clinical research plans.

## 1. Introduction

Since ocular pathologies often have no obvious symptoms in their early stages and are easily overlooked by patients, resulting in irreversible visual impairment of varying degrees by the time patients come to the clinic with ocular symptoms, routine screening, and early diagnosis of ocular diseases are critical [1, 2]. Meanwhile, the rich biological information of fundus images can reflect other tissues, organs, or systems and is expected to be applied. Therefore, the application of AI in fundus image classification, recognition, and semantic segmentation is expected to achieve large-scale screening and early diagnosis of ophthalmic diseases and improve the dilemma of lack of medical resources to a certain extent [3].

The first diagnostic methods of ophthalmic diseases were used by physicians to observe the structural morphology of the iris and pupil of the fundus using professional instruments such as biological ultramicroscopes, and then the observed images of the fundus structures were magnified and observed through visual field meters and atrial angioscopes, and various conditions and observations were integrated to diagnose whether the patient was suffering from an ophthalmic disease. Therefore, it can be seen that the traditional way of diagnosing ophthalmic diseases is complicated to operate and also requires a series of instrument tests to observe the patient, which takes a high time cost and makes the process of determining whether the patient has an ophthalmic disease more complicated.

At present, scholars at home and abroad mainly use machine learning and image processing and other technical methods to process fundus images, then combine the main contours and morphological changes of fundus images to detect the mutation characteristics of fundus images, and assist in the diagnosis of ophthalmic diseases, but there are not many studies using DL to detect ophthalmic diseases, and the research in this area is in a rapid development stage.

Increased intraocular pressure and hypertension are both current risk causes for the presence of ophthalmic diseases.  Figure 1 shows the basic structure of the fundus image.

The ocular structures of normal people include the ocular calyx, optic disc, macula, and arteriovenous system. The main site of eye diseases is the eye disc. The image below the eye contains a clear panel structure. Its color is mainly light red, orange, or white. It is the brightest area in the image below the eye because the light from it is reflected a lot. The optic disc consists of two important parts: the observation cup and the edge of the optic disc. The optic cup is in the center of the disc. The optic nerve bundle passes through the reticular disc and enters the cerebral cortex. Due to the pressure at the back, the physiological depression of the upper visual structure can be seen. After setting the visible cup, the edge of the optic disc represents the area between the viewing cup and the panel. When the visible ganglion cells die and fall to a certain extent, the visible cup changes, stretches, and contracts on the panel and finally changes the size of the two areas. This eventually led to the development of ophthalmic diseases.

## 2. Related Work

Although great strides have been made in the automatic diagnosis of diseases based on AI, the diagnostic results produced by such computer systems cannot be easily understood by doctors and patients. For example, some very simple visual observations that can be easily performed by humans are given to computers with unsatisfactory results. Some researchers have also made efforts in the interpretability of machine learning and have achieved some results. Reference [4] used decision trees to understand the choices made by support vector machines by combining the classification results of the support vector machines with the original sample feature vectors and then using the new data set to construct decision trees so that one can understand the classification logic. Reference [5] used deep belief networks that can be backward fixed retrospectively to understand the computer's rationale for autism diagnosis, and this study used human set features to discover what features are key factors in diagnosing autism. Reference [6] used the information to infer exactly which part of the image made the machine learning algorithm make such a classification decision while also facilitating human understanding of the classification results and the rationale for the classification. Reference [7] used masking tests to study the classification performance of DL algorithms after masking different parts of the image to trace the classification rationale and reasons for DL in a positive way. Reference [8] obtain the weight of each feature map by directly finding the derivative of the classification vector of the neural network with respect to the output of the convolution layer and later obtain a visual interpretation of the classification after multiplying and summing this weight with each feature map, which is a gradient-improved version of the literature.

Domestic scholars used two methods, mathematical morphology and Otsu's thresholding method, to determine the initial contour line of the fundus image, which solved the problems of poor adaptation of the fundus image and inaccurate edge localization, thus making the determined initial contour line closer to the optic cup of fundus image and making the segmentation rate of fundus image improved. By studying the multiphase active contour model, [9] made the optic disc of the fundus image take on an elliptical shape after the processing of the model and then completed the accurate segmentation of the optic disc by extracting the optic cup of the fundus image. Reference [10] proposed an algorithm to accurately localize the optic disc, which uses the direction of the vascular distribution of the fundus image to achieve the segmentation and localization of the optic disc. Reference [11] proposed using Markov random field theory so that the segmented fundus features can be used for the identification of ophthalmic diseases. Reference [12] proposed detecting the thickness of retinal nerve fibers by using the optical coherence tomography (OCT) technique to diagnose and treat patients with early ophthalmic diseases. Reference [13] proposed the use of a stacked sparse encoder for fundus image identification of ophthalmic diseases.

Foreign scholars [14] supplemented the image by first removing the blood vessels from the fundus image, using the top-hat transform, then segmenting the edge of the optic disc using the Hough transform method, and then applying the curve fitting method to extract to the exact region of the optic disc. Reference [15] proposed neural retinal rim ratio (NRR) as a parameter to perform aided diagnosis of ophthalmic diseases. Reference [16] proposed the use of Riemannian geometry to first analyze the fundus image before making an auxiliary diagnosis of ophthalmic diseases. Reference [17] proposed an adaptive deformation model to achieve diagnostic analysis of ophthalmic diseases. Reference [18] calculated the eigenvalues of fundus images for ophthalmic disease discrimination. However, the drawback is that the segmentation effect depends on the quality of fundus image acquisition [19]. Reference [20] determined the edges of the optic disc by a region growing algorithm and performed the cup-disc segmentation of fundus images by localizing the optic disc. Reference [21] proposed to make a determination of ophthalmic diseases by extracting and calculating the area and diameter of the fiber layer. Reference [22] proposed to classify fundus images of patients with early ophthalmic diseases, saving time for physicians to provide aid in the diagnosis, but the recognition rate needs to be improved.

In terms of interpretable machine learning for automatic diagnosis, [23] used the literature [24] and its gradient-improved version with intermediate volumes and feature maps generated using multiple deep convolutional neural networks to achieve interpretability of small sample medical images. Reference [25] collected intraoperative time series data of hemodynamic and ventilation parameters from more than 50,000 patients and achieved interpretable prediction of intraoperative hypoxia in patients with their own information and drug dose data, where interpretability is demonstrated by the importance of manually designed time series features.

Although the progress of these studies is remarkable, interpretable machine learning automated diagnostic platforms are rare, mainly because the design of these machine learning-based automated diagnostic methods does not follow human inertia, and interpretable DL ophthalmic diagnostic systems are even rarer.

## 3. Methods and Results

Currently, as medical technology has become better and better, researchers have designed a variety of equipment and instruments to screen for ocular diseases, through which the fundus images are acquired. The earliest of these devices was invented in 1851 by Hermann von Helmholtz, a German physician, who invented the fundoscope to observe the morphological structures of the fundus and thus diagnose ocular diseases by observing changes in the retina. Digital color fundus cameras and optical coherence tomography (OCT) are now commonly used in clinical practice for fundus image data acquisition.

The digital fundus camera can take pictures from different angles and record them in the form of digital images. For the identification of ophthalmic diseases in hospitals, the ophthalmologist usually adjusts the camera button manually to magnify and adjust the fundus area of the patient. The first is to determine the angle and type of shooting, normally adjusting the angle of the fundus camera between 30° and 55° and setting the type of shooting to dilate the diameter of the pupil to 5.5 mm or without dilating, with a pupil diameter greater than 3.3 mm. Next is the determination of the field of view; clinically, there can be four photographic fields of view: superior, temporal, inferior, and nasal; then there is refractive compensation, all ultimately to ensure that the clearest fundus image can be observed in the current state.

OCT was proposed by researchers at MIT in 1991 as a way to tomographically image a study subject by measuring the intensity of incident light. After more than 20 years of development and improvement, optical coherence tomography has become a tool for acquiring images with good camera results. Optical coherence tomography generates high-resolution fundus images by scanning the structures of the fundus.

OCT is now also available in most hospitals, but it is more expensive for patients to have a set of OCT examinations, and many patients choose the digital fundus camera examination method. Because of the low cost, rapid collection speed, and convenient storage of digital color fundus photography, fundus cameras are now widely used in various hospital ophthalmology examinations and have become a routine method of ophthalmology examination for patients, and the difficulty of collecting fundus images is much less than that of OCT images.

There are several network models in DL that are widely used. AlexNet, GooleNet, VGG-Net, and ResNet are some of the older network models, which were designed by Hinton and his students. The VGG-Net network is an improvement on AlexNet by increasing the depth of the network and shrinking the convolutional and pooling kernels. The ResNet network is used to redefine the channels by weighting the feature channels and using the useful image features to obtain a larger perceptual field. The M-ResNet network is designed to adjust the channel by using learning, redefine the channel features and fuse the features of the bottom layer and the top layer. The M-ResNet network completely takes into account the different features extracted from different layers and improves the learning and training capability of the network. The DL network structure M-ResNet designed in this paper is shown in Figure 2.

From Figure 2, it can be seen that the M-ResNet network has two stages: the first stage is the encoding stage, which inputs the image to the full convolutional layer. Since the features extracted by window sliding will cause the extracted feature information to overlap, the maximum pooling layer is used later to reduce the dimensionality and reduce the redundancy of convolution, and the maximum pooling layer does not cause bad segmentation accuracy of the image by compressing the image, which has little effect on the overall location region extraction later. The second stage is the decoding stage, where the compressed image is restored. The feature images extracted after the full convolution layer are restored to the same size of the image as in the encoding stage by the upsampling operation. The convolutional kernel sizes in the network are 1 × 1 and 3 × 3, both with a step length of 1. The nonlinear capability of the network is enhanced by adding the ReLU activation function after the fully connected layer, and the feature images are normalized by the BN layer after the convolutional layer, and the structure of M-ResNet is shown in Figure 3.

All examinees were photographed by the same examiner using a nondilated fundus color camera, and fundus photographs were taken with the macula as the center and the optic disc as the center. The patient was consulted by two fundus specialists, who independently performed 90D anterior microscopy under a slit lamp on the affected eye, and the diagnostic reports were obtained separately. The identical diagnostic results were taken as the final manual diagnosis, and in case of diagnostic discrepancies, the final diagnosis was determined by the chief ophthalmologist, and the above results were taken as the expert diagnosis group. The main diagnoses in this study included 14 diagnoses required for common clinical fundus diseases: (0) no significant abnormalities, (1) vitreous warts (outside the macula), (2) fundus arteriosclerosis, (3) age-related macular degeneration (ARMD) vitreous warts, (4) leopard-like fundus, (5) suspected cataract fundus/poor picture quality, (6) cup-to-disc ratio, (7) other macular degeneration, (8) macular anterior membrane, (9) other optic neuropathy, (10) unspecified abnormality – visit/observation, (11) large vitreous warts/pigmentation, (12) sporadic retinal hemorrhage, and (13) retina with medullary nerve fibers.

The first stage of this system process is the initial determination of the category to which the disease belongs, and in the research content of this chapter, there is no situation where multiple diseases appear in the compound, so this module is completed directly in the form of multiple classifications, and this module uses Inception-V4; in addition, the Inception-V4 models in the first stage are all used. The ImageNet data set pretrained model is initialized with convolutional layer weights and then fine-tuned. Its classification confusion matrix is shown in Figure 4. The classification accuracy was high for cataracts and lowest for normal human eyes, but in a practical application setting like hospitals, especially when applied for screening, false negatives are more important than false positives with a lower degree of risk. Also, the degree of confusion between pterygium and keratitis is higher. We analyzed the photos and found that pterygium and keratitis have some common symptoms, such as conjunctival congestion, and these image features made some misclassification by the neural network. Also, the error rate of keratitis and pterygium is relatively low, and the overall classification performance is excellent.

The second phase of the system was designed to achieve an important part of its interpretability, that is, to discriminate between different anatomical sites and important lesions in the ophthalmic slit-lamp images. This part of the experiment was completed using faster-RCNN, and the experimental procedure used quadruple cross-validation and was divided into two different faster-RCNN models responding to natural light slit-lamp photographs and cobalt blue light slit-lamp photographs. The specific difference mean accuracies of the cobalt blue light slit-lamp and localization results are shown in Tables 1 and 2 in the format of mean ± standard deviation, with a mean interpolation mean accuracy of 0.92 for identifying all categories in the cobalt blue light slit-lamp photo and 0.83 in the natural light cobalt blue light slit-lamp photo.

Figure 5 shows the results of the localization experiments corresponding to natural light sources. I–XV in Figure 5 represent the corneal iris region with keratitis, the keratitis lesion, the conjunctival sclera region, the corneal slit arc, the keratitis lesion slit arc, the eyelid, the iris slit arc, the congested scleral conjunctival region, the edematous conjunctival sclera region, the corneal iris region, the pterygium, the eyelid, the pupil region, the hemorrhagic conjunctival sclera region, and the cataract pupil region, respectively. The anatomic site definitions of keratoconjunctivitis are too fine, and some categories appear to overlap each other, which affects the experimental results, and these definitions are not taken into account in the actual clinical setting. In addition, the accuracy of eyelid localization is low. We analyzed the data source and found that the shape of the eyelid itself contains a certain curvature, so the rectangular box localization used here may not fit the shape of the eyelid very well, and more detailed image segmentation methods such as semantic segmentation are considered to cope with the eyelid in the subsequent work. Second, the eyelashes grow right on the eyelid, so the eyelid and eyelash regions also overlap. In addition, the faster-RCNN models in the second stage all use the ZF network pretrained with the ImageNet data set to initialize the convolutional layer weights.

The localization results for the four objects associated with the conjunctival-scleral zone (edema, congestion, hemorrhage, and normal conjunctival-scleral zone) were also unsatisfactory, mainly because the exposed part of the conjunctival-scleral zone also contains some curvature, but the rectangular target localization method used in this chapter was not able to fit this part effectively. In addition, the congested corneoscleral area shows some thickening and enlargement of the scleral vessels, but the details of these vessels may not be obvious under the convolutional neural network processing and may be confused with the normal conjunctival scleral area. Second, the edematous conjunctival scleral area is a three-dimensional structure, and it is difficult to distinguish this object from the two-dimensional planar images used in this chapter. Therefore, in future research, it may be necessary to put the detailed property determination of the conjunctival scleral zone in the third stage and use some simple image feature extraction and machine learning classifiers to avoid the overly coarse processing of CNN, such as LBP, color and texture features, and so on. The localization results of the pupillary area with cataracts were also not very good because the cornea is transparent, while the corneal iris area with keratoconus showed a white smoky appearance, and the cataract behaved very similarly to it, and the discrimination ability of faster-RCNN was reduced. Although there were poor localization results for some of the above objects, the overall localization results were satisfactory.

The third stage of the system is to determine the properties of each anatomical site and focal lesion in depth, with a total of 10 classification problems, of which problems 1–5, 6, 8, and 9 are dichotomous and the rest are triple classification problems. This module uses 50- and 101-layer residual neural networks with category weights and DenseNet to finely discriminate the attributes of each anatomical site and focal lesion, where the number of samples for each classification problem is shown in Table 3. This module is computed by intercepting all relevant site images according to the target localization in the second stage and then sending them to the residual network for classification to obtain the required information for refined clinical diagnosis. In addition, the residual network models in the third stage are fine-tuned by initializing the convolutional layer weights using the ImageNet dataset pretrained transfer learning model.

The performance metrics for the 10 classification problems in the third stage are in Table 4, where the format is mean ± standard deviation. For the three-classification problems, only the accuracy was counted; false positives and false negatives for the two-classification problems can be calculated by sensitivity and specificity, so they are omitted here. Their accuracy rates for all classification problems ranged from 0.79 to 0.98. The imbalance caused by the uneven data distribution in questions 2 and 5 is not mitigated by the treatment of the residual network with the addition of category weights, and the overall data sample size is sparse and difficult to expand.

After that, a 50-layer residual network was used for attribute determination of each anatomical site and focal lesion (see Table 5).

DenseNet with 121 layers was used to determine the attributes of each anatomical site and focal lesion, and its classification performance is in Table 6.

From the comparison of the experimental results of 50- and 101-layer residuals, the 50-layer residual network is better than the 101-layer residual network in alleviating the imbalance in the classification of imbalanced data sets, but for the amount of data in this module, more data supplementation is needed to more perfectly solve the imbalance results of individual classification problems in this module. Also, DenseNet cannot obtain good classification results in small samples. The ROC and AUC curves and precision-recall curves of the 101-layer residual network binary classification problems in the third stage of the system are shown in Figure 5. The overall performance of all binary classification problems is excellent.

Although the detailed attribute classification in the third stage depends on the target localization results in the second stage, the errors in the second stage have less impact on the third stage because the location information of the key anatomical sites required in the third stage are all located more accurately, including the corneal iris region with keratitis and the pterygium object.

In addition, the confusion matrix heat map for the two triple classification problems in the third stage of the system is shown in Figure 6. The experimental results showed good classification results for these two triple classification problems.

The ability of the 101- and 50-layer residual networks to process the complete photo input to distinguish the information needed for detailed diagnosis is verified here, and the performance of the 101- and 50-layer residual networks is shown in Tables 7 and 8, respectively.

From the experimental results, the classification results of the 101-layer residual network using the complete original image at the third stage are similar to those using the local anatomical site, while the classification results of the 50-layer residual network are much reduced. This means that the 101-layer residual network is better than the 50-layer residual network in finding the best result, that is, the 101-layer residual network is able to slowly clarify in the optimization process because of which part of the image this photo is classified as a certain class. However, it still cannot play the role of explanation.

The fourth stage of the system is the treatment decision based on the combined results of the first three stages, where the decision for pterygium is made by DL. The treatment plan for several other diseases can be obtained directly from the physician's questioning of the patient's condition combined with the results of the first three phases of the system. The logic is shown in Table 9. The factor of whether the pterygium has invaded the pupil or not is determined in this chapter by the aspect ratio of the pupil area localized in the slit-lamp photograph of the patient with pterygium disease, for example, if the aspect ratio deviates from 1 by a large amount, then the person's pupil has been invaded by the pterygium; otherwise, it is not.

The only pterygium that needs to be classified in the fourth stage is whether surgery is required using 101 layer residuals to complete, and the performance is shown in Figure 7, which is validated by the same quadruple cross-validation containing accuracy, sensitivity, and specificity. The second column shows the experimental results using the pterygium localization as input, and the third column shows the results using the complete original photograph as input. The localized input can effectively reduce the influence of other parts and reduce the useless noise input to enhance the classification performance.

## 4. Discussion

To conclude, in this study, the diagnoses of the included patients ranged from 1 to 5 (1.37 ± 0.68) diagnoses, and the accuracy of all diagnoses in the AI diagnostic group was 72.83%, of which the accuracy of only 1 diagnosis was 66.08%, 2 diagnoses were 77.97%, 3 diagnoses were 84.62%, 4 diagnoses were 96.00%. Among the results of only 1 diagnosis, 606 eyes (71.64%) had discrepancies due to leopard eye fundus diagnosis, and after removing the discrepancy of leopard eye fundus diagnosis, the accuracy of this group was 87.53%. This series of results illustrate the effectiveness of our proposed DL-based intelligent assisted diagnosis system for ophthalmic diseases.

## Figures and Tables

**Figure 1:** Fundus image structure.

**Figure 2:** M-ResNet network structure.

**Figure 3:** Structure of M-ResNet module.

**Figure 4:** Classification confusion matrix of the first phase of the system.

**Figure 5:** Classification ROC and precision-recall curves of the 101-layer residual network in the third stage of the system.

**Figure 6:** Heat map of the classification results for the two triple classification problems of the 101-layer residual network in the third stage of this system.

**Figure 7:** Performance of the system's fourth stage classification problem.

**Table 1:** Major target localization results in cobalt blue light slit-lamp photos.

Corneal iris area with keratitis		Keratoconus lesions	Corneal slit arc
1 ± 0		0.6748 ± 0.0503	1 ± 0
Keratoconus lesion slit arc	Iris fissure arc	Eyelid	Eyelash
0.8050 ± 0.1856	0.9658 ± 0.0781	0.9959 ± 0.0061	0.8579 ± 0.0059

**Table 2:** Main target localization results in natural light slit-lamp photographs.

Eyelash	Hemorrhagic conjunctival scleral area	Pupil area with cataract
0.6396 ± 0.0097	0.9084 ± 0.0013	0.8399 ± 0.0461
Eyelid	Edematous conjunctival scleral area	Normal conjunctival scleral area
0.8007 ± 0.0368	0.7405 ± 0.0647	0.7824 ± 0.0092
Pupillary area	Keratoconus lesion slit arc	Keratoconus lesion slit arc
0.8932 ± 0.0087	0.7227 ± 0.0998	0.8492 ± 0.0586
Iris fissure arc	Congested conjunctival scleral area	Corneal iris region
0.8176 ± 0.0343	0.6678 ± 0.0385	0.8610 ± 0.0517
Pterygium	Corneal iris area with keratitis	Keratoconus lesions
0.9756 ± 0.0445	0.9976 ± 0.0017	0.7625 ± 0.0583

**Table 3:** Data volume of each classification problem in the third stage of the system.

Question number	Data volume
1	Body hypertrophy: 157; body nonhypertrophy: 109
2	Pseudopterygium: 46; nonpseudopterygium: 220
3	Head augmentation: 170; head not augmented: 96
4	Head and body congested: 218; head and body uncongested: 48
5	Progressive phase:203: nonprogressive phase: 36
6	Corneal clouding invading the pupil area: 338; corneal clouding not invading the pupil area: 13
7	Infiltrative or ulcerative phase: 272; perforated phase: 48; healing phase with a quiet lesion (observation phase): 32
8	Corneal neovascularization: 176; corneal neovascularization not present: 175
9	Keratoconus lesion margin clear: 149; keratoconus lesion margin blurred: 204
10	Lamellar staining: 120; punctate staining or no staining: 25; corneal stump: 33

**Table 4:** Classification results of the third stage of this system using the 101-layer residual network.

Classification issues	Acc	Sensitivity	Specificity
1	0.7885 ± 0.0597	0.8961 ± 0.0391	0.7142 ± 0.0745
2	0.9648 ± 0.0296	0.7908 ± 0.1682	1 ± 0
3	0.7808 ± 0.0703	0.8716 ± 0.0939	0.6197 ± 0.1251
4	0.8852 ± 0.0150	0.9615 ± 0.0224	0.4998 ± 0.1172
5	0.9171 ± 0.0201	0.9821 ± 0	0.4687 ± 0.1574
6	0.9893 ± 0.0079	0.9883 ± 0.0169	0.9906 ± 0.0125
7	0.9805 ± 0.0142	—	—
8	0.9293 ± 0.0114	0.9483 ± 0.0391	0.9095 ± 0.0458
9	0.9342 ± 0.0443	0.9383 ± 0.0334	0.9315 ± 0.0726
10	0.9454 ± 0.0963	—	—

**Table 5:** Classification results of the third stage of this system using the 50-layer residual network.

Classification issues	Acc	Sensitivity	Specificity
1	0.8488 ± 0.0133	0.8763 ± 0.0431	0.7608 ± 0.0813
2	0.9768 ± 0.0201	0.8742 ± 0.0862	0.9954 ± 0.0096
3	0.7908 ± 0.0376	0.8739 ± 0.0345	0.642 ± 0.0963
4	0.9033 ± 0.0193	0.8838 ± 0.1708	0.5908 ± 0.1173
5	0.9147 ± 0.0151	0.9436 ± 0.0103	0.5000 ± 0.1022
6	0.9893 ± 0.0106	0.9851 ± 0.0178	0.9903 ± 0.6605
7	0.9745 ± 0.0097	—	—
8	0.9148 ± 0.0196	0.9192 ± 0.0614	0.9152 ± 0.0343
9	0.9085 ± 0.0392	0.9286 ± 0.0633	0.8554 ± 0.0997
10	0.9371 ± 0.0509	—	—

**Table 6:** Classification results of the third stage of the system using the 121-layer DenseNet.

Classification issues	Acc	Sensitivity	Specificity
1	0.6052 ± 0.0593	0.6075 ± 0.1877	0.7607 ± 0.0819
2	0.6453 ± 0.3275	0.3 ± 0.4765	0.7177 ± 0.4822
3	0.6589 ± 0.0539	0.8552 ± 0.1146	0.4131 ± 0.3065
4	0.7135 ± 0.1223	0.8379 ± 0.1483	0.2334 ± 0.2458
5	0.6139 ± 0.4462	0.6519 ± 0.4724	0.3425 ± 0.4782
6	0.6081 ± 0.0583	0.7587 ± 0.3231	0.5480 ± 0.3921
7	0.3906 ± 0.2115	—	—
8	0.6723 ± 0.0931	0.6903 ± 0.1077	0.6562 ± 0.2192
9	0.6841 ± 0.0560	0.5104 ± 0.2690	0.7273 ± 0.3369
10	0.6562 ± 0.1001	—	—

**Table 7:** Performance metrics for the third stage of the full classification problem using the original images (101-layer residual network).

Classification issues	Acc	Sensitivity	Specificity
1	0.8488 ± 0.0133	0.8769 ± 0.0534	0.7611 ± 0.0815
2	0.9768 ± 0.0202	0.8763 ± 0.0861	0.9964 ± 0.0096
3	0.7993 ± 0.0436	0.9739 ± 0.0345	0.6414 ± 0.0965
4	0.9033 ± 0.0191	0.9673 ± 0.0238	0.5908 ± 0.1175
5	0.9147 ± 0.0151	0.9436 ± 0.0103	0.5000 ± 0.1023
6	0.9893 ± 0.0106	0.9851 ± 0.0178	0.9903 ± 0.6605
7	0.9796 ± 0.0126	—	—
8	0.9148 ± 0.0196	0.9192 ± 0.0614	0.9152 ± 0.0343
9	0.9085 ± 0.0392	0.9286 ± 0.0633	0.8554 ± 0.0997
10	0.9154 ± 0.0963	—	—

**Table 8:** Performance metrics for the third stage of the full classification problem using the original images (50-layer residual network).

Classification issues	Acc	Sensitivity	Specificity
1	0.6668 ± 0.1483	0.5920 ± 0.4134	0.7186 ± 0.3171
2	0.8500 ± 0.0374	1 ± 0	0.1468 ± 0.2541
3	0.8125 ± 0.0779	0.9119 ± 0.0825	0.6756 ± 0.2605
4	0.7282 ± 0.1640	0.26 ± 0.6	0.8298 ± 0.3029
5	0.6095 ± 0.3356	0.7 ± 0.4203	0.6028 ± 0.4396
6	0.7047 ± 0.2035	0.9851 ± 0.0181	0.9903 ± 0.6605
7	0.4721 ± 0.2132	—	—
8	0.7234 ± 0.1521	0.5393 ± 0.3103	0.9137 ± 0.0898
9	0.8137 ± 0.0778	0.9119 ± 0.0825	0.7728 ± 0.0989
10	0.8776 ± 0.0695	—	—

**Table 9:** Logic of treatment recommendations for the fourth stage of the system.

	Surgery	Medication	Observation
Pterygium	Pupillary invasion (>1.5) or progressive stage or enlargement in the past 6 months	Congestion or bleeding in the head and body	
Subconjunctival hemorrhage		Congestion or hemorrhage	
Keratitis	Perforated phase or (quiet phase with corneal clouding) or ulcerated infiltrative phase >3 months	Ulcer infiltration or (quiet healing period, and <3 months) or photophobia and tearing	Quiet healing period and >3 months
Cataract	Cataract and (age >50 years or recent vision loss)		
Cobalt blue light slit-lamp	Perforated or near perforated	Lamellar staining	No staining or punctate staining

## Data Availability

The experimental data used to support the findings of this study are available from the corresponding author upon request.
